# Detection of COVID-19 Case from Chest CT Images Using Deformable Deep Convolutional Neural Network

**DOI:** 10.1155/2023/4301745

**Published:** 2023-02-16

**Authors:** Md. Foysal, A. B. M. Aowlad Hossain, Abdulsalam Yassine, M. Shamim Hossain

**Affiliations:** ^1^Department of Electronics and Communication Engineering, Khulna University of Engineering & Technology, Khulna 9203, Bangladesh; ^2^Department of Software Engineering, Lakehead University, Thunder Bay, ON, Canada; ^3^Department of Software Engineering, College of Computer and Information Sciences, King Saud University, Riyadh 11543, Saudi Arabia

## Abstract

The infectious coronavirus disease (COVID-19) has become a great threat to global human health. Timely and rapid detection of COVID-19 cases is very crucial to control its spreading through isolation measures as well as for proper treatment. Though the real-time reverse transcription-polymerase chain reaction (RT-PCR) test is a widely used technique for COVID-19 infection, recent researches suggest chest computed tomography (CT)-based screening as an effective substitute in cases of time and availability limitations of RT-PCR. In consequence, deep learning-based COVID-19 detection from chest CT images is gaining momentum. Furthermore, visual analysis of data has enhanced the opportunities of maximizing the prediction performance in this big data and deep learning realm. In this article, we have proposed two separate deformable deep networks converting from the conventional convolutional neural network (CNN) and the state-of-the-art ResNet-50, to detect COVID-19 cases from chest CT images. The impact of the deformable concept has been observed through performance comparative analysis among the designed deformable and normal models, and it is found that the deformable models show better prediction results than their normal form. Furthermore, the proposed deformable ResNet-50 model shows better performance than the proposed deformable CNN model. The gradient class activation mapping (Grad-CAM) technique has been used to visualize and check the targeted regions' localization effort at the final convolutional layer and has been found excellent. Total 2481 chest CT images have been used to evaluate the performance of the proposed models with a train-valid-test data splitting ratio of 80 : 10 : 10 in random fashion. The proposed deformable ResNet-50 model achieved training accuracy of 99.5% and test accuracy of 97.6% with specificity of 98.5% and sensitivity of 96.5% which are satisfactory compared with related works. The comprehensive discussion demonstrates that the proposed deformable ResNet-50 model-based COVID-19 detection technique can be useful for clinical applications.

## 1. Introduction

A massive outbreak of novel coronavirus disease (COVID-19) occurred in Wuhan, China, in December 2019, and it is causing a pandemic situation worldwide. According to the World Health Organization (WHO), around 476 million confirmed cases of COVID-19 including 6.1 million deaths were reported worldwide as of March 25, 2022 [1, 2]. The death rate is slightly less than 2%, but the main concern is the highly infectious nature of COVID-19 disease. The diagnosis of COVID-19 and isolation of patients are the most critical parts to control this pandemic situation. The mainstream diagnosis system is the real-time reverse transcription-polymerase chain reaction (RT-PCR) technique which is limitedly accessible to all hospitals and clinics. It also takes a long time to get the test results. The nucleic acid amplification testing (NAAT) is another technique for COVID-19 diagnosis which is also time consuming and exhibits low preciseness as reported in [3]. The chest imaging-based modalities such as X-ray (CXR) [4, 5], computed tomography (CT) [6–21], and ultrasound imaging [22, 23] are becoming popular alternatives to the pathological tests for not only accurate screening of COVID-19 cases but also for predicting the severity of the disease. Furthermore, recent studies show the promises of the medical image-based IoT healthcare framework for COVID-19 detection and social isolation suggestions through digital surveillance to deaccelerate the COVID spread [24–27]. Since a large amount of private information of patients is gathered in the IoT healthcare system for data fusion in COVID detection, a secured and protected system should be established for virtual medical facilities [28–31]. It is inevitable that the computer diagnosis is becoming an obvious and demanding support to the medical experts for proper diagnosis, prognosis, and treatment since the manual assessment of physicians is subjective in nature. Recent rapid advances of machine learning tools, especially deep learning, increase the power of computer-aided diagnosis significantly [32]. Therefore, the researchers are moving to diagnostic systems with medical imaging using machine learning technology because of its promises on testing results and severity analysis. Contextually, healthcare data visualization is of great importance for proper analysis, interpretation, and accurate prediction by highlighting the patterns, characteristics, and correlations. Therefore, in this big data and deep learning realm, the healthcare researchers and industries are emphasizing visual analysis of data in order to maximize the efficiencies of data-driven decisions and services.

In this study, chest CT scan images are used for COVID-19 detection due to its higher sensitivity than RT-PCR testing as demonstrated in [33]. The explicit form of the lungs and the presence of high rates of ground glass opacity (GGO) in COVID-19-infected lungs can be easily seen by CT scan images. Considering the proven extraordinary performance of recent deep learning techniques in computer-aided detection, we have employed a deep learning technique in CT images for detection of COVID-19 cases. Deep learning (DL) is just a class of machine learning (ML) in which multiple hidden layers are incorporated into the model to extract more complex features from input raw data. Nowadays, DL techniques have been successfully implemented in various fields such as image processing, image recognition and verification, network security, medical imaging, and healthcare.

There are lots of well-established deep convolutional neural network (CNN) architectures such as VGG16, ResNet-50, InceptionV3, and EfficientNet for object detection and classification tasks using images as input data. Last two years during the pandemic, various research works were conducted based on the DL method for COVID-19 classification, but to the best our knowledge the deformable CNN have not been used yet in this area. In this study, we have proposed two separate deformable deep convolutional networks considering the conventional CNN and the state-of-the-art ResNet-50 for COVID-19 detection from chest CT with a strategic emphasis on finding the impact of the deformable concept through a comparative performance analysis among the normal and deformable forms. The gradient class activation mapping (Grad-CAM) technique has been used to visualize and check the targeted regions' localizing effort at the final convolutional layer of the models. The main contributions of this work are as follows:

- Designing deformable convolutional neural network models in order to detect COVID-19 cases from chest CT images based on the conventional CNN and ResNet-50 architectures.
- Tuning the model to achieve superior performance and consequently training and validating it with a balanced dataset of COVID-19 chest CT images.
- Visual inspection of the localization capability of the convolution layers through Grad-CAM.
- Performance evaluation and inspection of the impact of deformable layers of the proposed models as well as comparative analysis with the related state-of-the-art techniques.

The rest of this article is organized as follows: A literature review of recent work is given in the related works section. The methodology section explains the proposed methodology as well as the model evaluation process. The next subsection presents the dataset used in this work, and the experimental result analysis has been explained in the experimental results and discussions section. Finally, the conclusion section concludes the whole research work.

## 2. Related Works

Numerous research works have been performed to diagnose COVID-19 from chest CT scan and X-ray images using ML and DL techniques. This section presents some recent studies related to COVID-19 detection from CT images applying DL techniques. A nine-layer tailored deep CNN model is proposed in [4] for COVID-19 screening using both CT and CXR images. They found the overall accuracy of 96.28% using a small dataset. Yasar and Ceylan [6] also proposed a deep CNN model with 23 layers, and it achieved the highest accuracy of 95.99%. Loey et al. [7] examined different well-known deep CNN architectures such as AlexNet, VGGNet16, and ResNet-50, utilizing the transfer learning technique for COVID-19 diagnosis using CT images. This work showed ResNet-50 can predict better than others with a test accuracy of 82.91%. Some work has been performed for segmentation as well as detection of COVID-19 using CT images in [8, 9], and they achieved accuracy of 94% and 94.67%, respectively. Ni et al. [8] proposed a combination of 3D U-Net and MVP-Net based architectures, whereas Amyar et al. [9] presented a method of the multitask learning architecture with an encoder and decoder system.

Singh et al. [10] designed a multiobjective differential mode-based CNN method for classification of COVID-19 cases, and their accuracy level is less than 93.5%. A machine-driven design exploration strategy-based deep CNN model is proposed for COVID-19 diagnosis in [11]. Wang et al. [12] designed a model by coupling two 3D U-Net architectures together for COVID-19 screening in CT images, and their classification accuracy reached 93.3%. A weakly supervised network is designed using the architecture ResNext+ along with the bidirectional LSTM blocks for prediction of COVID-19 cases from volume and slice-level CT images in [13].

Ensemble learning is now becoming a popular technique because of its higher precision and accuracy instead of using a single model. Several studies implemented an ensemble of transfer learning using different pretrained deep neural network architectures such as VGG, Xception, and ResNet for screening COVID-19 cases. Aversano et al. [14] exploit the transfer learning technique by using pretrained models such as VGG, Xception, and ResNet individually and then combining to have an ensemble model. Their experiment shows the value of *F*1-score ranges from 0.94 to 0.95. Gifani et al. [15] used 15 pretrained standard CNN models to build an ensemble architecture with the majority voting rule with experimental results showing the overall detection accuracy of 85.4%. Biswas et al. [16] also proposed an ensemble of deep transfer learning using VGG16, ResNet-50, and Xception models for CT image classification with good accuracy. In our previous study, we have developed an ensemble model for COVID-19 screening from CT images, exploiting three deep CNN architectures in [17]. The experimental results achieved the accuracy of 96% and a sensitivity of 97% for CT scan image prediction.

After reviewing the above research works, it is concluded that the deep learning method can be employed for COVID-19 screening purposes though there were some limitations such as imbalanced datasets and high rates of false prediction. So there is still a scope to improve the prediction accuracy more as well as the robustness of the methods that can minimize the false positive and false negative rates. In this work, we proposed a deep learning approach for COVID-19 detection using CT images. A deformable technique is implemented in the standard ResNet-50 architecture to make the model more robust by replacing a few layers of ResNet-50 with its deformable parts to achieve the good prediction performance.

## 3. Methodology

This section covers mainly three parts of the methodology for COVID-19 detection: (a) describing the idea of the deformable CNN, (b) explaining the proposed framework using the deformable concept, and (c) mentioning different evaluation criteria to validate the proposed framework. Description of the CT scan dataset used in this researh is provided at the end of this section. 

### 3.1. Deformable CNN

The standard CNNs are limited in their ability to model complex geometric transformations due to their fixed geometric composition of modules. The convolution kernel selects the samples at fixed spatial location, and the pooling layer reduces the spatial resolution at a constant ratio in regular CNN modules. As a consequence, it reduces the effectiveness of models for complex transformation. So the adaptive determination of sampling locations or deformed kernels based on the objects is required for exact visual recognition. In this regard, Dai et al. [34] introduced a new approach of deformable convolutional neural networks which was done at Microsoft Research Asia in 2017. They introduced two new modules to enhance the capability of transformation modeling: deformable convolution and deformable ROI pooling. Deformable convolution adds a 2D offset to sampling locations of regular convolution grids to deform the kernel in an adaptive manner based on the required objects.

Let a convolutional kernel of *S* sampling locations, *w*_*i*_ and *l*_*i*_ denote the weight and offset for the *i*-th location of the kernel, respectively. Then, *y*(*l*) denoting the output features from the input feature *x*(*l*) at location *l* is calculated as follows:

(1) $$\begin{array}{c} y\left(l\right)=\overset{S}{\underset{i=1}{\sum }}w_{i}∙x\left(l+l_{i}\right)\text{.} \end{array}$$

For deformable convolution, equation (1) will be

(2) $$\begin{array}{c} y\left(l\right)=\overset{S}{\underset{i=1}{\sum }}w_{i}∙x\left(l+l_{i}+∆l_{i}\right)\text{,} \end{array}$$

where the standard grid of *S* sampling locations is augmented with offsets *∆l*_*i*_ which is a learnable offset. As *l* + *l*_*i*_ + *∆l*_*i*_ is now fractional, bilinear interpolation is used to calculate *x*(*l* *+* *l*_*i*_ + *∆l*_*i*_) in equation (2) [34]. The kernel geometric structure of the deformable convolution system is illustrated in Figure 1.

The offsets for kernel deformation are obtained by standard back-propagation of the gradients with the bilinear interpolation operations during training of the model. An additional convolution layer is used to learn the offset values shown in Figure 2. As a consequence, a small amount of parameters is added to the model for offset learning. In another study [35], it is proved that the performance can be enhanced by stacking more deformable layers in standard CNN architectures. So taking these benefits of deformable CNNs, we employed this idea for COVID-19 detection.

### 3.2. Proposed Model

A deformable convolution concept is utilized in this work for the detection of COVID-19 cases from chest CT images. We have designed two separate deformable deep convolutional networks considering the conventional CNN and the state-of-the-art ResNet-50 for the detection task. The strategic emphasis is to observe the influence of the deformable concept through a comparative performance analysis between the normal and deformable forms. Initially, a fifteen-layered deep CNN model is developed, and then its deformable form is created. Deformable form of this normal CNN model is made by replacing two convolution layers with deformable convolution layers. The detailed layers and parameter information of both normal and deformable CNN models are shown in Table 1. Before selecting this fifteen-layered model, we have experimented with various architectures by tuning different parameters of the models and also the position of deformable layers to find the best performance. Then, this fifteen-layered structure is chosen for COVID-19 detection in CT images on the basis of the maximum performance. It is seen that the total number of parameters of the deformable model is greater than the normal CNN model as some extra parameters are needed for offsets learning in the deformable convolution. Every convolution layer uses the ReLU activation function except the final dense layer that uses softmax activation for binary classification.

The overfitting and underfitting problems are the common problems inducing in the deep learning model. These problems are also addressed carefully in our experiments. The dropout layer with a drop rate of 0.4 is used in each model to diminish the overfitting problems. A large dataset is used to train the models to overcome the underfitting problems. Also, the number of layers in the models and training epochs is increased after tuning the models to solve the underfitting problems. The performances of these models are presented in the results section.

To make the COVID-19 classification task more robust and effective, we proposed a state-of-the-art CNN architecture, ResNet-50, with its deformable format which is shown in Figure 3. It contains five convolutional stages followed by a final fully connected dense layer for classification. Stages 2 to 5 have uniform convolutional (ConvBlock) and identity blocks (ID_Block) in the regular ResNet-50. Each convolutional and identity block contains a skip connection which is first introduced in the ResNet model and is the main strength of the ResNet architecture. Two of the standard Conv2D layers in the second stage convolutional block of ResNet-50 are replaced by the corresponding deformable convolution layers (Deform_Conv2D) to form a deformable convolutional block (Deform_ConvBlock). The detailed architectures of each block are also presented in Figure 3. Then, it is formed as the deformable CNN or deformable ResNet-50.

The ResNet-50 architecture is selected in the CT image classification task due to its notable performance that is proved by the different state-of-the-art medical imaging research [7]. Due to its skip connection, it is easy to train the deep network, and the deeper the network, the more suitable it is for medical image classification. The ResNet architectures have the capability to solve the vanishing gradient problems due to their identity mapping systems. So, this robust ResNet-50 model can be effectively used for COVID-19 screening. In this work, this ResNet-50 model is created from the scratch as its defined architecture; no pretrained weights are used for classification. The positions of the deform layers are fixed after extensive tuning of the model for best performance. The ReLU function is used as activation in each layer except the final layer which uses softmax activation for binary prediction.

As stated, additional parameters are needed in the deformable CNN model to learn the offsets of the kernel's deformed position. So the proposed deformable ResNet-50 model requires more parameters than the regular ResNet-50 model. The total number of parameters in the proposed model is 23,771,906, whereas the regular ResNet-50 model contains 23,591,810 parameters. The extra 180,096 parameters actually used for deformation learning tasks in the proposed model make it more robust and stronger. Hence, the proposed method presented in Figure 3 can be one of the most efficient ways of COVID-19 screening using lung CT images.

### 3.3. Evaluation Criteria

The commonly used assessment metrics for DL classification models are utilized to assess the proposed methodology. The metrics are accuracy, specificity, sensitivity, *f*1-score, and precision measured in terms of true and false prediction values. As only accuracy metrics cannot show the effectiveness of deep learning models for classification, various ways of assessment are used in this study. Besides these metrics measurement, the accuracy and loss curves with the number of epochs have also been analyzed for performance evaluation. Equations (3)–(7) represent the definitions of accuracy (Acc), specificity (*S*_*p*_), sensitivity (*S*_*n*_), *f*1-score (*F*_*s*_), and precision (*P*_*r*_), respectively.

(3) $$\begin{array}{c} Acc=\frac{tp+tn}{tp+tn+fp+fn}\text{,} \end{array}$$

(4) $$\begin{array}{c} S_{p}=\frac{tn}{tn+fp}\text{,} \end{array}$$

(5) $$\begin{array}{c} S_{n}=\frac{tp}{tp+fn}\text{,} \end{array}$$

(6) $$\begin{array}{c} F_{s}=\frac{2\times tp}{2\times tp+fp+fn}\text{,} \end{array}$$

(7) $$\begin{array}{c} P_{r}=\frac{tp}{tp+fp}\text{,} \end{array}$$

where the true positive (*tp*) and true negative (*tn*) denote the value of correct predictions of actual COVID positive patients and non-COVID patients, respectively. False positive (*fp*) and false negative (*fn*) denote the value of incorrect predictions of COVID positive and negative patients, respectively. The confusion matrix is also utilized to show the value of true and false predictions in a comfortable way of visualization which is shown in Figure 4.

### 3.4. Dataset Description

CT scan images have a detailed and clear view of the lungs as compared to CXR images. So it is a very convenient way to diagnose the COVID-19 disease using CT images. A chest CT scan dataset is collected from the kaggle dataset repository for this experiment of COVID-19 diagnosis. The CT images of this dataset have been collected from different real patients in hospitals from Sao Paulo, Brazil [36]. It contains a total of 2481 CT images, including 1252 images for COVID-positive patients and 1229 images for non-COVID cases with other lung diseases. The main symptom of COVID-19 in CT is the two-sided existence of irregular ground glass opacities (GGOs) that may merge into dense and consolidative lesions beneath the pleura and along the bronchovascular networks. The number and area of the lesions increase with the disease's progression. Furthermore, beside the GGOs patterns such as interstitial widening, crazy-paving pattern, halo and reversed halo patterns, airway and vascular modifications are also found in CT for COVID-19 cases [37]. Few sample COVID and non-COVID CT slices from this dataset are shown in Figure 5.

The collected CT dataset is almost a balanced dataset which is an important factor of the model learning phase in the deep CNN. An imbalanced dataset may mislead the output prediction in deep learning classification tasks. In this experiment, no preprocessing techniques are applied due to irregular opacification present in CT images of pulmonary diseases. So raw CT scans are used for COVID-19 detection purposes because preprocessing can cause the loss of actual sensitive information about the texture of the infected region.

## 4. Experimental Results and Discussions

All the experiments were performed on the Google colaboratory platform using the Keras and Tensor Flow libraries. The programs were run on GPU with 12.69 GB RAM and 107.72 GB Disk provided by Python-3 Google compute engine backend. In total, four experiments were performed in this study, consisting of a fifteen-layered CNN with its normal as well as deformable form and a ResNet-50 model with its normal as well as deformable form for COVID-19 screening.

Both the normal and deformable fifteen-layered CNN models are trained and validated using the collected COVID-19 CT dataset with input shapes of 150 × 150 × 3. The dropout rate of 0.4 is used in the dropout layer of both configurations. The Adam optimizer with the learning rate of 0.001 and the categorical cross-entropy loss function are employed to compile the models. The number of epochs and other hyperparameters are tuned for the best learning process. Finally, the number of epochs is selected as 60. The train-valid-test splitting ratio is used as 80 : 10 : 10, and Figure 6 shows the learning curves of both the normal and deformable CNN.

The erratic nature is seen from the model accuracy curve due to the raw CT images of random passing to the models shown in Figure 6. In the training phase, callback is utilized for saving the best model with the highest accuracy. The training accuracy reached 91.8% and 90.3% in the normal and deformable CNN, respectively. Then, the models are saved with validation accuracies of 90.7% and 91.9% for the normal and deformable CNN, respectively. Finally, the models are tested independently with a test dataset which is 10% of the main dataset splitted initially. The test accuracy of 92.4% and 93.2% have been found in the normal and deformable CNN, respectively. The confusion matrixes are exhibited in Figure 7 for the analysis of true and false predictions. It is expected that the deformable model can minimize the overall false prediction. So, from Figure 7 the overall false prediction value is reduced in the deformable CNN model. This experiment shows the deformable CNN can outperform the regular CNN.

Then, the state-of-the-art CNN model, ResNet-50, has been selected for this experiment of COVID-19 screening. Primarily, the whole model has been developed from scratch, according to its original architecture. Then, its deformable form is created as mentioned in the proposed model subsection. All the parameters of both models (normal ResNet-50 and proposed deformable ResNet-50) are trained through the collected CT dataset; no transfer learning technique is employed here. The training dataset has been selected for learning the model with input shapes of 64 × 64 × 3. The hyperparameters are selected to the standard value after various tuning processes addressing overfitting and underfitting problems. The Adam optimizer and categorical cross entropy loss function are used to compile the normal ResNet-50 and deformable ResNet-50 models. The learning curves for both normal and deformable ResNet-50 models are shown in Figure 8. Though a sudden abrupt shifting is seen in the learning phase of models as in Figure 8(b), the callback function is used in these experiments to get the best model with higher accuracy. The training accuracy in the proposed deformable ResNet-50 model reached 99.5%. The ratio between validation and test datasets was the same as in the previous experiments. Both the normal and deformable parts of the ResNet-50 model are saved with the validation accuracy of 95.2% and 95.6%, respectively. Finally, the normal and proposed deformable ResNet-50 models have been tested with the test dataset. The test accuracies have been reached at 96.8% and 97.6% for normal ResNet-50 and proposed deformable ResNet-50, respectively. It shows the best performance of the proposed deformable ResNet-50 model.

The confusion matrixes for both regular ResNet-50 and proposed deformable ResNet-50 models are shown in Figure 9. The total number of false predictions is reduced from 8 to 6 in deformable ResNet-50. From this confusion matrix, it is clear that the proposed deformable ResNet-50 model is more robust and strengthened than its regular form.  Table 2 represents the overall test results of four experiments in this study. According to Table 2, the accuracy of deformable experiments has superior results as compared to their base counterparts. Each of the four models has been tested with a single CT image by loading the model with trained weights. All the experiments can give the appropriate prediction result within a few milliseconds by inputting a single CT scan image.

Computation time is an important factor for model performance analysis and for any diagnosis system. In this regard, we have calculated the CPU times required for a single CT image prediction in all our experiments. CPU times depend on the input image shape. For the first two experiments (the normal and deformable fifteen-layered CNN), input image shapes were 150 × 150 × 3 and then the regular and proposed deformable ResNet-50 took input shapes of 64 × 64 × 3. The normal and deformable fifteen-layered CNN take CPU times of 46.7 ms and 71.6 ms, respectively, for the prediction of a single CT image. This time includes image loading and resizing according to the model's input shape and then prediction. Then, the normal ResNet-50 model and the proposed deformable ResNet-50 model take CPU times of 55.2 ms and 68.1 ms, respectively, for a single image. Hence, the deformable part takes little more time than its original form due to the extra parameters contains in deformable parts.

The receiver operating characteristics (ROC) curve is a widely used graphical representation of classifier performance.  Figure 10 illustrates the ROC curve for all experiments, including our proposed method. It shows the area under curve (AUC) values of all models. The AUC is found to be 0.998 from the ROC curve for the proposed deformable ResNet-50 model, and it indicates the effectiveness of our proposed method for COVID-19 detection.

The Grad-CAM visualization is a useful tool for differentiating the model learning capability in positive and negative cases using the heatmap view in the images [38]. It uses gradients of the final convolutional layer to distinguish the region of interest for a specific class.  Figure 11 shows the Grad-CAM view of (a) COVID images (Class 1) and (b) non-COVID images (Class 0) produced by the proposed method. In Figure 11(a), ground glass opacity and consolidation of the COVID-infected lungs are accurately highlighted by the green color that indicates the good sensitivity of the model. In Figure 11(b), no specific opacity or consolidation is detected in CT images due to the negative cases, and it shows the dispersed green colors in the images. Therefore, viewing the Grad-CAM, it can be mentioned that the convolutions layer framework-based feature extractor of the proposed deformable ResNet-50 model is well supported as the classifier input.

In this study, we have also discussed comparative analysis with the related deep learning-based state-of-the-art works. Most of the time, the performance metrics of deep learning models depend on the size of the dataset used for training. So the articles that used the same dataset or one that was close to our employed dataset size as well as related deep CNN models were selected for appropriate comparison of performances.  Table 3 presents the comparative analysis of the detection results with the recent works. As it is seen from Table 3, results of the proposed deformable ResNet-50 model outperform the related methods. It also shows very low false predictions as it has the model geometric deformation capability. So, it can be a reliable and useful technique for the clinical application of COVID-19 screening.

## 5. Conclusions

The deployment of DL techniques in the various medical diagnosis systems is now growing worldwide, and it speeds up the early diagnosis system in healthcare environments. In this article, we have proposed a COVID-19 disease detection technique from chest CT using the deformable deep CNN. Different experiments were performed for better model selection. The impact of the deformable concept has been examined through performance comparative analysis among the designed deformable and normal models, and it is found that the deformable models show better prediction results than their normal form. Extensive analysis shows that the proposed deformable ResNet-50 model performs satisfactorily with an accuracy of 97.6% compared with the state-of-the-art techniques. The Grad-CAM visualization evidences of the targeted regions' localizing tendency at the final convolutional layer is also found noteworthy. In the future, more diverse and critical CT datasets will be utilized for training to boost the robustness of the model. Finally, this study showed that the proposed method can be useful for effective COVID-19 detection as a substitute for RT-PCR with time and availability limitations.

## Figures and Tables

**Figure 1:** Kernel geometric structure of the deformable convolution process: (a) standard 3 × 3 convolution grid points, and (b) sampling locations (red dots) after deformable convolution.

**Figure 2:** Illustration of deformable convolution with 3 × 3 kernel.

**Figure 3:** The architecture of the proposed deformable ResNet-50 model.

**Figure 4:** The confusion matrix.

**Figure 5:** Sample CT slices from the dataset (a) for COVID cases and (b) for non-COVID cases.

**Figure 6:** Training accuracy curves for (a) the normal CNN and (b) the deformable CNN.

**Figure 7:** Confusion matrixes for the prediction of (a) the normal CNN and (b) the deformable CNN.

**Figure 8:** Training accuracy curves for (a) normal ResNet-50 and (b) proposed deformable ResNet-50.

**Figure 9:** Confusion matrixes for the prediction of (a) normal ResNet-50 and (b) proposed deformable ResNet-50.

**Figure 10:** ROC curves for all experiments with AUC values.

**Figure 11:** Grad-CAM visualization for (a) class 1 (COVID) and (b) class 0 (non-COVID).

**Table 1:** Summary of the proposed deformable deep CNN and its base normal CNN.

Deformable CNN		Normal CNN	
Layers	Output shape	Layers	Output shape
Input layer	[150, 150, 3]	Input layer	[150, 150, 3]
Conv 2D	[148, 148, 16]	Conv2D	[148, 148, 16]
Batch normalization	[148, 148, 16]	Batch normalization	[148, 148, 16]
Max pooling 2D	[74, 74, 16]	Max pooling 2D	[74, 74, 16]
**Deform conv 2D**	**[74, 74, 16]**	Conv 2D	**[74, 74, 16]**
Conv 2D	[72, 72, 32]	Conv2D	[72, 72, 32]
Max pooling 2D	[36, 36, 32]	Max pooling 2D	[36, 36, 32]
**Deform conv 2D**	**[36, 36, 32]**	Conv 2D	**[36, 36, 32]**
Conv 2D	[34, 34, 64]	Conv2D	[34, 34, 64]
Max pooling 2D	[17, 17, 64]	Max pooling 2D	[17, 17, 64]
Dropout	[17, 17, 64]	Dropout	[17, 17, 64]
Flatten	[18496]	Flatten	[18496]
Dense	[256]	Dense	[256]
Dropout	[256]	Dropout	[256]
Dense	[2]	Dense	[2]
Total parameters **4,764,098**		Total parameters **4,761,154**	

The bold terms are the main focus of our proposed deformable CNN architecture.

**Table 2:** Performance results of all experiments.

Models	Accuracy (Acc)	Specificity (*S*_*p*_)	Sensitivity (*S*_*n*_)	*F*1-score (*F*_*s*_)	Precision (*P*_*r*_)
15-layered normal CNN	0.924	0.919	0.929	0.917	0.905
15-layered deformable CNN	**0.932**	0.882	0.991	0.929	0.875
Normal ResNet-50	0.968	0.971	0.965	0.965	0.965
Deformable ResNet-50 (Proposed)	**0.976**	**0.985**	**0.965**	**0.973**	**0.982**

**Table 3:** Comparative analysis of classification results with recent related studies.

Study	Method	Performance		
		Acc (%)	*S*_*p*_ (%)	*S*_*n*_ (%)
Yasar and Ceylan [6]	23-layer deep CNN	95.9	99.0	94.0
Amyar et al. [9]	Multitask DL (with the encoder and the decoder)	94.6	92.0	96.0
Wang et al. [12]	3D-ResNets	93.3	95.5	87.6
Sun et al. [18]	AFS-DF	91.7	89.9	93.0
Hasan et al. [19]	DenseNet-121	92.0	—	—
Wang et al. [20]	Modified inception V3	89.5	88.0	87.0
Cai et al. [21]	ResNet-18	94.3	97.3	91.4
Proposed	Deformable ResNet-50	**97.6**	**98.5**	**96.5**

## Data Availability

In this research, the dataset is collected from kaggle dataset repository [36]. The dataset is publicly available at https://www.kaggle.com/datasets/plameneduardo/sarscov2-ctscan-dataset.

## References

[1] (2022). WHO coronavirus (COVID-19) dashboard. https://covid19.who.int.

[2] (2019). Report of the WHO-China joint mission on coronavirus disease (COVID-19). https://www.who.int/publications/i/item/report-of-the-who-china-joint-mission-on-coronavirus-disease-2019-(covid-19).

[3] Xie C., Jiang L., Huang G. (2020). Comparison of different samples for 2019 novel coronavirus detection by nucleic acid amplification tests. *International Journal of Infectious Diseases*.

[4] Mukherjee H., Ghosh S., Dhar A., Obaidullah S. M., Santosh K. C., Roy K. (2020). Deep neural network to detect COVID-19: one architecture for both CT Scans and Chest X-rays. *Applied Intelligence*.

[5] Shorfuzzaman M., Hossain M. S. (2021). MetaCOVID: a siamese neural network framework with contrastive loss for n-shot diagnosis of COVID-19 patients. *Pattern Recognition*.

[6] Yasar H., Ceylan M. (2020). A novel comparative study for detection of COVID-19 on CT lung images using texture analysis machine learning and deep learning methods. *Multimedia Tools and Applications*.

[7] Loey M., Manogaran G., Khalifa N. E. M. (2020). A deep transfer learning model with classical data augmentation and CGAN to detect COVID-19 from chest CT radiography digital images. *Neural Computing & Applications*.

[8] Ni Q., Sun Z. Y., Qi L. (2020). A deep learning approach to characterize 2019 coronavirus disease (COVID-19) pneumonia in chest CT images. *European Radiology*.

[9] Amyar A., Modzelewski R., Li H., Ruan S. (2020). Multi-task deep learning based CT imaging analysis for COVID-19 pneumonia: classification and segmentation. *Computers in Biology and Medicine*.

[10] Singh D., Kumar V., Kaur M., Kaur M. (2020). Classification of COVID-19 patients from chest CT images using multi-objective differential evolution-based convolutional neural networks. *European Journal of Clinical Microbiology & Infectious Diseases*.

[11] Gunraj H., Wang L., Wong A. (2020). COVIDNet-CT: a tailored deep convolutional neural network design for detection of COVID-19 cases from chest CT images. *Frontiers of Medicine*.

[12] Wang J., Bao Y., Wen Y. (2020). Prior-Attention residual learning for more discriminative COVID-19 screening in CT images. *IEEE Transactions on Medical Imaging*.

[13] Mohammed A., Wang C., Zhao M. (2020). Weakly-Supervised network for detection of COVID-19 in chest CT scans. *IEEE Access*.

[14] Aversano L., Bernardi M. L., Cimitile M., Pecori R. (2021). Deep neural networks ensemble to detect COVID-19 from CT scans. *Pattern Recognition*.

[15] Gifani P., Shalbaf A., Vafaeezadeh M. (2020). Automated detection of COVID-19 using ensemble of transfer learning with deep convolutional neural network based on CT scans. *Int. J. CARS*.

[16] Biswas S., Chatterjee S., Majee A., Sen S., Schwenker F., Sarkar R. (2021). Prediction of COVID-19 from chest CT images using an ensemble of deep learning models. *Applied Sciences*.

[17] Foysal M., Aowlad Hossain A. B. M. COVID-19 detection from chest CT images using ensemble deep convolutional neural network.

[18] Sun L., Mo Z., Yan F. (2020). Adaptive feature selection guided deep forest for COVID-19 classification with chest CT. *IEEE Journal of Biomedical and Health Informatics*.

[19] Hasan N., Bao Y., Shawon A., Huang Y. (2021). DenseNet convolutional neural networks application for predicting COVID-19 using CT image. *SN Comput. Science*.

[20] Wang S., Kang B., Ma J. (2021). A deep learning algorithm using CT images to screen for Corona virus disease (COVID-19). *European Radiology*.

[21] Cai X., Wang Y., Sun X., Liu W., Tang Y., Li W. Comparing the performance of ResNets on COVID-19 diagnosis using CT scans.

[22] Muhammad G., Shamim Hossain M. (2021). COVID-19 and non-COVID-19 classification using multi-layers fusion from lung ultrasound images. *Information Fusion*.

[23] Nouvenne A., Zani M. D., Milanese G. (2020). Lung ultrasound in COVID-19 pneumonia: correlations with chest CT on hospital admission. *Respiration*.

[24] Hossain M. S., Muhammad G., Guizani N. (2020). Explainable AI and mass surveillance system-based healthcare framework to combat COVID-I9 like pandemics. *IEEE Network*.

[25] Shorfuzzaman M., Hossain M. S., Alhamid M. F. (2021). Towards the sustainable development of smart cities through mass video surveillance: a response to the COVID-19 pandemic. *Sustainable Cities and Society*.

[26] Kamruzzaman M. M., Alrashdi I., Alqazzaz A. (2022). New opportunities, challenges, and applications of edge-AI for connected healthcare in internet of medical things for smart cities. *Journal of Healthcare Engineering*.

[27] Yassine A., Hossain M. S. (2022). COVID-19 networking demand: an auction-based mechanism for automated selection of edge computing services. *IEEE Transactions on Network Science and Engineering*.

[28] Lin H., Garg S., Hu J., Wang X., Jalil Piran M., Hossain M. S. (2021). Privacy-enhanced data fusion for COVID-19 applications in intelligent Internet of Medical Things. *IEEE Internet of Things Journal*.

[29] Masud M., Gaba G. S., Alqahtani S. (2021). A lightweight and robust secure key establishment protocol for internet of medical things in COVID-19 patients care. *IEEE Internet of Things Journal*.

[30] Rahman A., Hossain M. S., Alrajeh N. A., Alsolami F. (2021). Adversarial examples-security threats to COVID-19 deep learning systems in medical IoT devices. *IEEE Internet of Things Journal*.

[31] Hossain M. S., Muhammad G. (2018). Emotion-aware connected healthcare big data towards 5G. *IEEE Internet of Things Journal*.

[32] Yanase J., Triantaphyllou E. (2019). A systematic survey of computer-aided diagnosis in medicine: past and present developments. *Expert Systems with Applications*.

[33] Ai T., Yang Z., Hou H. (2020). Correlation of chest CT and RT-PCR testing for coronavirus disease 2019 (COVID-19) in China: a report of 1014 cases. *Radiology*.

[34] Dai J., Qi H., Xiong Y. (2017). Deformable convolutional networks. https://arxiv.org/abs/1703.06211.

[35] Zhu X., Hu H., Lin S., Dai J. Deformable ConvNets v2: more deformable, better results.

[36] Soares E., Angelov P., Biaso S., Froes M. H., Abe D. K. (2020). Sars‐cov-2 CT‐scan dataset: A large dataset of real patients CT scans for sars‐cov-2 identification, medRxiv.

[37] Carotti M., Salaffi F., Sarzi-Puttini P. (2020). Chest CT features of coronavirus disease 2019 (COVID-19) pneumonia: key points for radiologists. *Radiologia Medica, La*.

[38] Selvaraju R. R., Cogswell M., Das A., Vedantam R., Parikh D., Batra D. (2020). Grad-CAM: visual explanations from deep networks via gradient-based localization. *International Journal of Computer Vision*.

